RETRACTED

# A hybrid PSO-FFNN approach for optimized seismic design and accurate structural response prediction in steel moment-resisting frames

**DOI:** 10.1371/journal.pone.0322396

**Published:** 2025-06-02

**Authors:** Qiong Liu

**Affiliations:** College of Finance and Economics, Yinchuan University of Science and Technology, Yinchuan, Ningxia, China; SRMIST (Deemed to be University): SRM Institute of Science and Technology (Deemed to be University), INDIA

## Abstract

The first steel is the most prevalent material used in building. Steel’s intrinsic hardness and durability make it appropriate for different uses, but its greater adaptability makes it ideal for seismic design. The brittle fracture occurred in welded moment connections of steel structures, which were originally thought to be ductile for resistance to earthquakes. The research aims to optimize structural parameters in steel structure seismic design. This paper presents an effective technique for the best seismic design of steel structures, which consists of two computational methodologies. First, particle swarm optimization (PSO) was presented to accurately define the structural characteristics in the seismic design of steel constructions, then a feed-forward neural network (FFNN) to determine unconventional seismic design methodologies for steel frameworks, precisely forecast the structural responses, and improve seismic resistance and dependability under dynamic conditions by using high-tech components and technological advancements. This study presents designing a realistic storey steel moment-resisting frame (MRF) structure and maximum weight under full seismic loading. The outcome demonstrates the reduction in generations that was accomplished during the optimization procedure. Although the PSO method in the paper converges in lower generations, the process indeed requires a significant amount of computing power. The FFNN approach involves the suggestion of a neural network model that works well to predict the necessary structural reactions during optimization. The proposed model considerably minimizes the total computation time. Study aims to improve the seismic analysis of steel using PSO along with forecasting structural responses using a network of feed-forward neural networks (FFNN) to enhance accuracy and reduce the computation time (2.4 min). The proposed FFNN model is more accurate than earlier methods, with the lowest MAPE values in S_IO (3.0661), S_LS (3.562), and S_CP (3.9252). Moreover, it reveals the highest predictive precision with the lowest RRMSE values of 0.0231 (S_IO), 0.0281 (S_LS), and 0.0314 (S_CP). Moreover, the FFNN model has a competitive run time of 2.4 minutes while possessing good goodness-of-fit, with 1.0096, 1.0995, and 0.9925 of R2 for S_IO, S_LS, and S_CP, respectively. As compared to WCFBP-RB, the proposed PSO+FFNN model has better prediction for S_IO, where the predicted value of 0.7879 is almost identical to the actual value of 0.8000. As compared to WCFBP-RB, the model predicts 1.4085 for S_LS, while the actual value is 1.4388. For S_CP, PSO+FFNN predicts 1.8621, which is more precise than WCFBP-RB and almost equals the actual figure of 1.9000.

RETRACTED

## 1. Introduction

Excessive deformation in buildings can be avoided when they are designed according to seismic regulations, thereby preventing failure and ensuring occupant safety during earthquakes. One key factor in assessing post-earthquake structural integrity is Residual Interstory Drift (RID), which results from the plastic deformation of structural components during seismic events. When comparing the costs of retrofitting versus repairing buildings after seismic excitation, the RID ratio is a crucial parameter to consider [1]. To conduct numerical simulations, modern architectural and engineering models for complex and nonlinear structures primarily rely on computational methodologies. One of the most widely used simulation-based methods for dynamic structural modeling is Nonlinear Response History Analysis (NRHA), often in conjunction with finite element analysis. These methodologies have applications in various fields, including thermal transfer, fluid flow, electromagnetic potential, and structural analysis [2]. In steel plate-based damping systems integrated within moment-resisting frames (MRFs), stiffness defines the structure’s ability to resist bending under applied forces. Several factors influence this stiffness, including the length, width, material composition, and connection details of steel plates. Unlike adaptability, stiffness is typically measured as rigidity, which affects the damper’s overall performance [3]. Additionally, the elasticity and flexibility of steel structures influence how forces are distributed across metal plates, impacting both structural dispersion and geometric design considerations.

Despite advancements in seismic analysis, no prior research has specifically focused on the accuracy of forecasting seismic drift effects in steel moment-resisting frames [4]. However, conducting highly detailed NRHA simulations for large-scale regional seismic assessments is often impractical due to computational limitations [5]. Optimization techniques have proven useful in overcoming the computational challenges associated with seismic analysis and steel frame design. Several researchers have explored the application of metaheuristic algorithms to improve both linear and nonlinear seismic response evaluations [6]. Additionally, in the field of structural health monitoring (SHM) and damage recognition, machine learning (ML) techniques have been recently adopted to identify damage-sensitive parameters [7]. These ML-driven model updating strategies refine initial structural models to more accurately represent damaged buildings [8]. A promising innovation in seismic damping systems is the development of S-shaped steel dampers, which exhibit distinct hysteretic properties. While cement-reinforced structures are a well-established construction method, they possess low axial load capacity and limited vertical flexibility, particularly in high-rise buildings and heavily loaded bridges [9]. To address these limitations, metal-strengthened concrete alloys have been introduced, incorporating embedded steel components to enhance load-bearing capacity and adaptability.

RETRACTED

Seismic forces exert significant energy on structures, often leading to severe damage [10]. Consequently, rapid and reliable seismic performance evaluation methods are essential for effective retrofitting and reuse strategies [11]. This study aims to investigate seismic design strategies for steel structures, leveraging network-based simulations and optimization techniques. A key focus is on Moment-Resisting Frames (MRFs), which are widely used for resisting lateral forces (e.g., wind and earthquakes) through rigid beam-column connections. These frames offer high ductility and flexibility, making them a preferred solution for earthquake-resistant structures. Accurate seismic design can minimize inordinate deformation in structures, ensuring both the safety of occupants and structural integrity during earthquakes. RID, an essential parameter in measuring post-earthquake structural condition, is the result of plastic deformation in the structural elements. While considering retrofit costs vs. repair costs after seismic activities, RID plays a vital role. Computational methods, including NRHA in association with finite element analysis, have become more important in modern physics since they are increasingly used to study complex and nonlinear structural systems. Issues like stochastic loadings, irregular response factors, and nonlinear material characteristics have become simpler to manage, thanks to the enhanced computing capacity.

This research is unique in that it integrates optimization and predictive modeling within one framework by integrating Particle Swarm Optimization (PSO) with a Feed-Forward Neural Network (FFNN) to optimize seismic design parameters for steel structures. With a computation time of just 2.4 minutes, this hybrid method significantly enhances the precision of seismic response prediction. By achieving the minimum MAPE (3.0661–3.9252) and RRMSE (0.0231–0.0314) values out of all the parameters (S_IO, S_LS, and S_CP), the proposed FFNN model has better performance than conventional methods. With R2 values ranging as high as 1.0995, the model also illustrates great goodness-of-fit, presenting excellent predictive reliability. The PSO+FFNN model tends to make forecasts closer to the true seismic reactions compared to WCFBP-RB.

RETRACTED

### Contributions of the study

- Paper introduces a revolutionary technique for optimizing structural parameters in steel structures using FFNN and PSO.
- Effectiveness of PSO in discovering optimal parameters for structure for steel frameworks under seismic loading, resulting in fewer generations required for convergence.
- Technique FFNN is used to reliably predict structure responses, increasing the dependability of seismic design forecasts.
- Apply the proposed approaches to a six-story steel MRF to demonstrate practical application.

Study’s subsequent sections are organized as follows. Part 2 deals with related works. The methods are explained in Part 3. The result is shown in Part 4. Section 5 offers the conclusion.

## 2. Related works

Fang et al. [12] proposed the DBN by architecture was utilized in the functioning of cold-rolled metal channel segments with edge-stiffened/unstiffened systemic pores under axial compression. Using a model of linear regression generated by Paddle, it was observed that the huge training set using the suggested DBN fared better than both approaches. Li et al. [13] suggested a methodology to improve the effectiveness of assessing structure seismic reactions, which was based on the ensemble machine learning paradigm. The efficiency with which structural parameters were determined during the initial design phase might be greatly increased by that suggested methodology, which would cut down on the number of trail evaluation iterations. Van der Westhuizen et al. [14] suggested a new formulation that takes into consideration the soil-structure interaction effect as well as various architectural aspects of the superstructure that the dissertation study focused on applying machine learning methods and the connection found during the validation phase demonstrated the high predictive characteristics for steel frameworks. A model-based technique that combines the use of a continuous wavelet transformation of the response signal with a CNN was also referred to evaluate the health of the steel organization linkage by Paral et al. [15]. With just global vibration data based on impulsive stimulation on the structure required for the approach, a better finite-element model for the steel framework that considers interconnection flexibility can be employed for a range of purposes, as expressed by Wang et al. [16]. The shear resistance model was created using a variety of ML techniques that have partial dependency plots to provide a reasonable explanation for the elements influencing the shear strength. An enormous-scale steel plane frame’s estimated ideal kinds and brace locations can be extracted using a method that has been given. Seismic loads were applied to the frame, and restrictions on the maximum strain in the framework elements were determined by the type of bracing used in every story and the greatest inters Tory drift angle was suggested by Sakaguchi et al. [17]. Building a surrogate model can significantly lower the processing expenses for architectural evaluation throughout the procedure of optimization. Naser et al. [18] opened up new avenues for research and motivated the community to use contemporary technology to achieve effective and cutting-edge design solutions. Non-iterative model linearization methods created compact, one-step predictive phrases that can precisely forecast the dimensional responses of concrete-filled steel tubes columns. These algorithms include computational genetics and gene expression programming. Building frame brace location has been approached using a simulated annealing used machine learning to identify suboptimal alternatives during refinement was suggested by Bond et al. [19]. To define the features that characterize the solutions and minimize the number of variables, both pooling and convolution were employed. Synthetic annealing, a form of heuristics based on local exploration, was used to carry out optimization and results in seismic design for steel frameworks to enrich steel goods. The impairment locating technique described to identify the input frame of steel photos as damaged or undamaged steel parts in employed a network of DCNN by Kim et al. [20]. The DCNN-DL approach was used for the real-time examination and localization of steel frame deterioration, as the research demonstrated. Han et al. [21] used a labelled picture set of damaged matrix pictures to train the second version of the mobile deep learning model. CNNs and time-frequency domain analysis were utilized to locate lateral support problems in various steel construction components. The results suggest that combining deep learning techniques with time-frequency analysis could improve the accuracy of locating the compromised steel frame support components. De Rezende et al. [22] was to advance the fields of artificial intelligence and SHM by showcasing yet another possible use for CNN in supporting the ISHM method for diagnosing structural damage in spinning machinery. To do this, the structural strength of a rotor consisting of two bearings with balls, two storage mechanisms, and one shaft was monitored while accounting for four different functioning speeds and three various medical conditions. Following Table 1 provides the research gap among the existing studies.

RETRACTED

**Table 1:** Research gap.

Author	Proposed Technique	Significance	Limitations
Fang et al. [12]	Deep Belief Network (DBN) for cold-rolled metal segments under axial compression	Improved performance with large training set compared to other methods	Limited to axial compression of cold-rolled metal segments
Li et al. [13]	Ensemble Machine Learning for seismic response assessment	Enhanced efficiency in determining structural parameters, reduced trial iterations	Specific to early-stage seismic response evaluation
Van der Westhuizen et al. [14]	ML model considering soil-structure interaction	High prediction accuracy for steel frameworks	Focused mainly on steel frameworks, may not generalize
Paral et al. [15]	CNN + Continuous Wavelet Transform for health monitoring	Evaluates steel structure health using only global vibration data	Requires impulsive stimulation data
Wang et al. [16]	Finite Element Model + ML for shear resistance	Explains shear strength influencing factors using partial dependency plots	Focused on shear resistance, limited by input data quality
Sakaguchi et al. [17]	ML-based surrogate model for brace optimization	Reduces computational cost in optimization process	Limited to specific brace types and seismic loading conditions
Naser et al. [18]	Gene Expression Programming for concrete-filled steel tubes	Accurately forecasts dimensional responses, encourages innovative design methods	Specific to concrete-filled steel tubes
Bond et al. [19]	Simulated Annealing + ML for brace location optimization	Identifies suboptimal brace locations during design refinement	Relies on heuristic optimization, may miss global optimum
Kim et al. [20]	Deep Convolutional Neural Network (DCNN) for damage detection in steel frames	Real-time detection and localization of steel frame deterioration	Requires labeled images for training
Han et al. [21]	Mobile DL model + CNN + Time-Frequency Analysis for lateral support issues	Improves accuracy in detecting lateral support problems in steel structures	Focused on lateral support, may need diverse datasets
De Rezende et al. [22]	CNN for diagnosing damage in rotating machinery within SHM framework	Supports ISHM by monitoring rotor health under various speeds and conditions	Limited to rotating machinery, not general to all structures

RETRACTED

## 3. Methodology

The use of modern techniques provides earthquake safety and resilience and includes choosing appropriate materials, creating ductile frames, and using inventive connecting features to withstand seismic stresses, thereby reducing damage and guaranteeing the structure’s strength during and after seismic occurrences Design variables, ground velocity, many constraints, numerous design parameters, quantity a matrix, encoding matrix, persistence matrix, to precisely determine the structural features involved in the seismic analysis of steel constructions and the PSO optimizes the following structural parameters of time, velocity vectors, displacement vector information, unit vector, non-dimensional ratio of component categories, inter-storey drift ratios, penalty operation, adjusting factor, and objective function and the Natural Periods, Non-Dimensional Ratios of Component Teams, Inter-Storey Drift The ratios (x and y direction) To precisely forecast the structural response, the following data are classified into the FFNN model which has ground movement data, design variables, time points, displacement vector data, velocity vector, element the group attributes, load and boundary conditions, response spectra, environmental variables, and material properties. Research utilizes ground motion data and design variables together with time points and displacement and velocity vector data and element group attributes as its input factors. Response spectra and inter-story drift ratios (x and y directions) together with boundary conditions, loads and material characteristics and environmental conditions and non-dimensional element group ratios were incorporated. Structural responses were optimized and their predictions done using the goal function together with penalty function and adjusting factor.The data mentioned above is presented in S1 Table.

### 3.1 Optimal seismic design problem

The process of solving the following optimization formulation to determine the design variables is known as the optimal layout of structures that experience seismic loading in Equations (1–4).


$$W;W_{j}\in Q^{d};j=1,\;.\;.\;.\;,\;m$$ (1)

e(w) (2)

$$h_{i}\left(\dot{W}.Y(s),\dot{Y}(s),\ddot{Y}(s),s\right)\leq 0;i=1,\ldots ,n$$ (3)

$$N\ddot{Y}(s)+D\dot{Y}(s)+LY(s)-NJ{\ddot{v}}_{h}(s)=0$$ (4)

The following factors are critical in time-variant optimization problems: quantity matrix(N), encoding matrix(D ), durability matrix(L), ground velocity (${\ddot{u}}_{g}$(t)), numerous limitations(m), number of design parameters (n), time(s), velocity vector (${\dot{Y}}_{s}$), displacement vector data(Y(s)), unit vector(J), and number of design variables vector(W). There is a finite value set ($Q^{d}$) available. Throughout the optimization process, variance and non-dimensional relation requirements, which are critical for stability and performance, are taken into consideration, guaranteeing that system responses stay within reasonable bounds as performed in Equations (5–7).


$$\mathrm{\backslash [}h_{l}(W,s)=\frac{c_{k}(W,s)}{c_{l,all}}-1\leq 0;l=1,\ldots .,mt\mathrm{\backslash ]}$$ (5)

$if\frac{e_{bk}(W,s)}{E_{b}}\leq 0.15:$


$$\mathrm{\backslash [}h_{k}(W.s)-1=\frac{e_{bk}(W,s)}{E_{b}}+\frac{e_{azk}(W,s)}{E_{az}}+\frac{e_{ayk}(W,s)}{E_{ay}}-1\leq 0;k=1,\ldots ,mf\mathrm{\backslash ]}$$ (6)

$if\frac{e_{bk}(W,s)}{E_{b}}>0.15:$


$$\mathrm{\backslash [}h_{k}(W,s)=r_{k}(W,s)-1=\frac{e_{bk}(W,s)}{E_{b}}+\frac{D_{nz}e_{azk}(w,s)}{\frac{\left(1-e_{bk}(W,s\right)}{{E^{\prime }}_{fz}})E_{az}}+\frac{D_{ny}e_{ayk}(w,s)}{\frac{\left(1-e_{bk}(W,s\right)}{{E^{\prime }}_{fy}})E_{ay}}-1\leq 0\;h_{k}(W,s)=r_{k}(W,s)-1\frac{e_{bk}(W,s)}{0.6E_{z}}+\frac{e_{azk}(W,s)}{E_{az}}+\frac{e_{ayk}(W,s)}{E_{ay}}-1\leq 0\;\mathrm{\backslash ]}$$ (7)

The total number of elements, nodes, and deviation values for the $L_{th}$stories are indicated by (mf), (mt), and ($c_{k}$) in theseismic analysis for steel structures, respectively. (azk)Represents the compressive axial stress, ($E_{az}$) and ($E_{ay}$) represent the bending loads about wand saxes of the $k_{TH}$ element, respectively. ($e_{bk}$), ($F_{b}$), ($e_{azk}$), and ($e_{ayl}$) are acceptable values for these parameters. One of the most important design factors for ensuring structural performance and safety during seismic occurrences is the yield stress, or$E_{z}$ suggests in Equation (8).


$$\mathrm{\backslash [}D_{nz}=D_{ny}=0.85,\;aslo,{E^{\prime }}_{fz}=\frac{{12\pi }^{2}F}{23{\left(l_{z}k_{z}/q_{z}\right)}^{2}}and{E^{\prime }}_{fy}=\frac{{12\pi }^{2}F}{23{\left(l_{y}k_{y}/q_{y}\right)}^{2}}\mathrm{\backslash ]}$$ (8)

Finding the actual length factor (l) is necessary for estimating permissible radial and Euler stresses in seismic analysis for steel structures and this study uses estimated explicit calculations for un-braced frames. These formulas offer useful approximations for(l), making computations in seismic design more efficient. They can utilize these streamlined formulas to ensure that structural components meet both performance and safety standards under seismic loads, finding a compromise between accuracy and efficiency in seismic design conditions employed in Equation (9).


$$\mathrm{\backslash [}L=\sqrt{\frac{1.6H_{B}H_{A}+4\left(H_{B}+H_{A}\right)+7.5}{H_{B}+H_{A}+7.5}},\;H=\frac{\sum \left(\frac{J_{d}}{K_{d}}\right)}{\sum \left(\frac{J_{h}}{K_{h}}\right)}\;\mathrm{\backslash ]}$$ (9)

The suffixes A and B represent the position of endpoints in seismic evaluation for steel constructions. Moments of inertia are represented by${\;(j}_{d}$) and ($j_{h}$), and the suspended lengths of beams and columns are denoted by ($K_{d}$) and ($K_{h}$). The symbol ∑1 represents the total of every component joined at an intersection in the bending plane. The seismic design code of UBC is used in this work. The maximum rigid reaction dispersion (Δm) in each story is calculated based on these factors by UBC drift control regulations to guarantee the integrity of the structure under seismic loading shown in Equation (10).

$\Delta_{N}=0.7{Q\Delta }_{t}$ (10)

The behavior factor is indicated by (R) in the seismic structure design of steel buildings and the torsional distortion of each story is represented by (Δt), both of which need to be assessed at all structurally significant points. P-Δ effects must be considered in the study to compute the maximal rigid responsive displacement, (ΔN). To ensure an appropriate assessment of the structure’s performance under seismic conditions, ($c_{1}(W,s)$) shows in Equation (11) is derived taking these effects into account. This method makes sure that the effects of structural deformations as well as the initial elasticity response are appropriately taken into account.


$$\mathrm{\backslash [}c_{l}(W,s)=\frac{\Delta_{Nl}(W,s)-\Delta_{Nl-1}(W,s)}{g_{l}}\mathrm{\backslash ]}$$ (11)

$$=\frac{0.7\left(\Delta_{Tl}(W,s)-\Delta_{Tl-1}(W,s)\right)}{g_{l}};l=1,\ldots ,mt$$

Analysis of time history should be used to calculate the response of systems subjected to seismic loads. This study focuses on developing computer software using the Newmark method. Because every barrier in the seismic design is time-dependent, overcoming them with a large computing cost. This study takes a standard way of dealing with time-dependent restrictions. This approach divides the period into ($T_{l})$ segments and applies limitations at each time grid point. This method ensures an accurate assessment of limitations during seismic occurrences for seismic designs. The computation for the $l_{th}$ time limit is as follows: this enables a full examination of structural performance under various earthquake stresses, ensuring strong design and conformance to safety rules in Equation (12).


$$h_{i}\left(W,Y\left(s_{\alpha }\right),\;\dot{Y}\left(s_{\alpha }\right),\ddot{Y}\left(s_{\alpha }\right),s_{\alpha }\right)\leq 0,\;\alpha =0,\ldots ,mo$$ (12)

A time range ($s_{i}$) is used for implementing restrictions in seismic design is split into ($h_{i}$) subintervals and as a result, reliable estimation of structural performance during the seismic event is ensured by evaluating the time-dependent constraints at (gl+1) time grid positions employs in Equation (13).


$$e(W)=\{e(W)ifW\in \tilde{\Delta }\;e(W)+e_{o}(W)otherwise\;$$ (13)

After performing a seismic check on the structure, the limiting every time grid point allows for the evaluation of a function. Following that, the aim functionality for optimal seismic design is defined, with a focus on lowering structural reactions and ensuring safety while adhering to seismic performance criteria throughout the analysis.


$$e_{o}(W)=\sum_{\alpha =0}^{m_{ho}}q_{o}[\;\sum_{k=1}^{mf}(\max(h_{k}\left(W,s_{\alpha }\right){,{0))}^{2}+\;\sum_{l=1}^{mt}({\left(h_{l}\left(W,s_{\alpha }\right),0\right)}^{2}+\varepsilon ]}^{0}$$ (14)

Where $q_{o},$ ∆~, and $\left(e_{o}W\right)$ stand for the penalty function, an adjustment factor, and the possible search space, in that order and the following term ε defines the small positive number o prevent undefined behavior when the bracketed term is 0.

RETRACTED

### 3.2 Define the structural characteristics in the seismic design of steel organizations using particle swarm optimization

Validation of PSO implementation must include established benchmarks which prove its efficiency and its effectiveness in structural optimization tasks. Standard optimization algorithms including Genetic Algorithms and Differential Evolution and Ant Colony Optimization should serve as benchmarks against which the performance of PSO can be assessed. Tests performed on established structural engineering problems and optimization tests help evaluate PSO models through the measurement of their speed of convergence solution quality and computational expenditure. This verification process confirms that PSO delivers competitive reliable solutions for designing steel frameworks under seismic loading relative to recognized methods used in the engineering field.

PSO is used in structural characteristics in the seismic design of steel structures and they are started at random in the optimization field of search problem by the number of design parameters, quantity matrix, encode a matrix, durability matrix, grounding velocity, and several limitations Time, speed vector, displaced vector data, unit vector, and velocity vector Non-dimensional Element Group Ratio, The PSO optimizes these structural parameters to precisely characterize the structural properties in the seismic analysis of steel constructions. The parameters that are used in the steel framework seismic design are Inter-Storey Drift Ratios, Penal Function, Adjusting Factor, and Objective Function and the optimization to lessen the design’s computational load. Every swarm particle exhibits potential. In PSO, every solution variable is given that the problem should be converted from a discrete form to an integer that represents the cross-section number. The positions of the particles are modified as they traverse across the search space, taking into account each iteration’s best individual particle placements. The optimal location in the search space is found by evaluating the perceived fitness of the particles. The swarm is updated using the subsequent relations at each optimization in Equations (15 and 16).


$$u_{j}^{l+1}={\omega u}_{j}^{l}+d_{1}q_{1}\left(o_{j}^{l}-w_{j}^{l}\right)+d_{2}q_{2}\left(o_{h}^{l}-w_{j}^{l}\right)$$ (15)

$$w_{j}^{l+1}=w_{j}^{l}+u_{j}^{l+1}$$ (16)

Where the present positioning vector ($w_{j}^{i}$) and the $i_{th}$particle’s velocity vector $u_{j}^{i}$at the ${j\;}_{th}$iteration, correspondingly where, d1 and d2 are constants. This parameter creates the PSO, which is improved as follows$(O_{h}$) is the pre-eminent global point between all the particles in the swarm, also known as the global ideal; q1 and q2 are dual equally scattered random values taken from the (0, 1) domain; and v is an inaction mass cast-off to discount the particle’s previous speed. During a run, the acceleration weight is typically thought of as a linearly declining function that ranges from 0.9 to 0.4. In this work, Equation (16) is modified in Equation (17) to improve the PSO’s exploration capability.


$$w_{j}^{l+1}=w_{j}^{l}+e(u_{j}^{l+1},o)$$ (17)

Where f is an expected value “O” specified and an exponential coefficient ($u_{j}^{i+1}$) was expressed in Equation (18).


$$e\left(u_{j}^{l+1},o\right)=\{round\left(u_{j}^{l+1}\right)u_{j}^{l+1}\geq 1\;1\;u_{j}^{l+1}<1\;ando\leq rand\;1\;u_{j}^{l+1}<1\;ando>rand\;$$ (18)

Where a consistently distributed random value from the (0, 1) domain is called a rand. In this case, the rounding function is represented by round (.), and “**O**” equals 0.2. Because the problem at hand involves a discrete area, the function only rounds the velocity vector to boost the exploration rate throughout iterations. Stated otherwise, the enhancement increases the algorithm’s likelihood of exploring its search space in next rounds.

RETRACTED

PSO algorithm demonstrates exceptional capability in finding best parameters for steel frameworks which experience seismic loading. Through simultaneous exploration and exploitation PSO optimizes the search of complex design spaces and reaches convergence in fewer generations. The optimization performance improves significantly with reduced computational time thanks to PSO when compared with traditional procedures and makes this technique optimal for dynamic loading applications. The physical meaning of optimization constraints within structural engineering needs better integration with their usage in the current study. The structural system’s safety along with its serviceability and cost-effectiveness receives direct impact from three constraints that include member size limitations and inter-story drift as well as load-carrying capacity restrictions. The presentation currently fails to provide direct connections between constraints applied in the study and actual structural engineering demands like seismic ability and building regulation requirements. The research would achieve better practical applicability by providing a comprehensive analysis of how the constraints modify optimization results as well as enhance steel framework integrity and seismic performance.

### 3.3 Prediction of structural responses using Feed – Forward Neural Network (FFNN)

FFNNs utilize the seismic analysis of steel constructions and the prediction of structural responses uses the parameters such as Non-Dimensional The ratios of Element Teams, Inter-Storey Drifting Rates (x and y orientations), Time points, displacement vector data, design variables, load and boundary conditions, element group properties, response spectrums, conditions in the environment, and material properties are all included in the ground motion data set. Input layer, which is equal to the network inputs; Nand M neurons make up the initial and subsequent hidden layers, respectively one neuron makes up the resultant layer. A variety of time points, acceleration and movement vectors, element properties, and ambient circumstances constitute the input data for the structural analysis (Fig 1). The structural responses to various loads and boundary conditions are evaluated using this information. After processing these inputs, the model indicates whether the structural response is critical/unsatisfactory (expressed by 1) or non-critical (represented by 0). Based on the provided data, the result shows if the structural reaction satisfies safety and performance requirements. The FFNN model was employed due to its ability to accurately predict structural performance properties under complex loading conditions by capturing highly non-linear relationships between input and output variables. Regression problems, like those encountered in structural engineering applications, are highly advantaged by its flexibility in handling large datasets and detecting intricate patterns. Moreover, FFNNs are well-suited to this research application because they have been rigorously tested in similar studies with consistent convergence, strong generalization, and adaptability to varying input variables.

RETRACTED

**Fig 1:** Feed-forward neural network.

A linear being enabled function serves as the output transfer function, and the sigmoid utility serves as the transferral mechanism for the concealed neurons. The following Equation (19) is used to determine the j^th^ hidden neuron’s output.


$$\mathrm{\backslash [}z_{i}=\frac{1}{\left[1+f^{-(\sum_{j=1}^{m}(x_{ij}w_{j}-a_{i}))\;}\right]}i=1,2,\ldots ,M\mathrm{\backslash ]}$$ (19)

The data input layer contains numerous cells that use FFNN that is proportional to the total number in the steel network inputs there are N and  M cells in the first and second submerged layers, respectively and there is only one neuron in the resultant layer. A linear being enabled function serves as the output transfer function and the sigmoid function is used as a value of transfer for hidden neurons. The following formula is used to determine the $j_{th}$hidden neuron’s output was expressed in Equation (20).


$$\mathrm{\backslash [}y_{l}=\frac{1}{\left[1+f^{-(\sum_{j=1}^{M}(x_{li}z_{i}-a_{l}))\;}\right]}l=1,2,\ldots .,N\mathrm{\backslash ]}$$ (20)

Where $(x_{i})i_{th}$is input, ${(y}_{j})$ is the output, and ($x_{j}^{i})$is the quantity of weight the distance between the$i_{TH}$layer of input and the $j_{th}$first hidden neuron. This is the location of the first concealed layer. The resulting Equation (21) finds the subsequent hidden layer$\left(z_{k}\right)$.


$${PO}_{k}=\sum_{l=1}^{N}\left(x_{kl}y_{l}\right)k=1,2,\ldots ,G$$ (21)

Where ($x_{kl}$) denotes the total weight of the $K_{TH}$output neuron and the $l_{th}$subsequent hidden neuron. By calculating the disparity between the expected output and the FFNN output the efficiency of assessment of the original training algorithm. The mean square error (MSE) is calculated in this case:


$$NTF=\frac{1}{m}\sum_{j=1}^{m}{\left({PO}_{j}-S_{j}\right)}^{2}$$ (22)

Where ${(s}_{j})$ is the target output, $\left({PO}_{j}\right)$ is the output that was received from the FFNN, andn is the overall total of training patterns. The training is calculated using the following Equation (23) result’s fitness value.


$$Fitness\left(W_{j}\right)=Min.(NTF)=Min\left[\frac{1}{m}\sum_{j=1}^{m}{\left({PO}_{j}-S_{j}\right)}^{2}\right]$$ (23)

The MSE via the goal output and the expected result from the FFNN is minimized using the back-propagating algorithm’s decreasing gradient. The biases and weights of the steel are taken from the resultant layer are updated toward the hidden layers using the Mean Squared Error (MSE) here’s how the revised weights are calculated in Equations (24 and 25).


$${\Delta \omega }_{ij}=\gamma (z_{i}-w_{j})$$ (24)

$${\Delta a}_{i}=\left(z_{i}-w_{j}\right)$$ (25)

Where gis the learning rate,$({\Delta a}_{i}$) is an alteration in bias, and $\left({\Delta \omega }_{ij}\right)$ is the variation in the weight of the steel that links the inputs of the first hidden neurons. Next, the revised biases and weights are provided as thereafter Intriguing ¼ bold þ shows in Equations (26 and 27).


$$a_{new}=a_{old}+\Delta a$$ (26)

$$\omega_{new}=\omega_{old}+\Delta \omega$$ (27)

To obtain the necessary accuracy, it is crucial to choose appropriate input variables for the multi-task single-task learning framework built on the FFNN model. Three input parameters are utilized to generate the FFNN model and$S_{IO},S_{LS}$,$S_{CP}$ as well as the temperature of the steel particle in seismic designs.

RETRACTED

## 4. Results

The data set employed for the optimization of structural parameters in seismic design using the PSO algorithm is comprised of 5,000 samples, which are randomly sampled from experimental and simulated data. Of these, 3,500 samples (70%) were dedicated to training, 1,000 samples (20%) to validation, and 500 samples (10%) to testing. The database contains necessary structural parameters like beam and column sizes, bay spacing, and story height, as well as material properties like steel grade, yield strength, and modulus of elasticity. Further, seismic load parameters like the base shear coefficient, inter-story drift ratio, and damping ratio were included to analyze structural performance. Response measures like maximum displacement, residual drift, and energy dissipation efficiency were also documented. The process of random selection guarantees diversity in structural configurations, and thus the dataset is apt for training strong predictive models for seismic optimization.

Study improves seismic design variables for structural steel employing FFNN and PSO. PSO effectively detects structural parameters, whereas FFNN forecasts structural responses, resulting in faster calculation and higher accuracy. Paper illustrates good earthquake design, emphasizing the fewer generations required for optimizing with PSO. The layout of a 6-story steel skyscraper focuses on maximizing earthquake resilience. Key features include using flexible steel materials, creating deformable MRF, and using modern computational tools to forecast and improve the strength of the structure, ensuring stability and security during seismic events while preserving the design and functional integrity in Fig 2.

**Fig 2:** Architectural design of 6-storey steel structures.

Table 1 shows the efficiency of models based on neural networks (WCFBP-RB, WCFBP-PW1, WCFBP-MH [23] and FFNN (Proposed) in predicting seismic reactions for six-story steel structures. MAPE, RRMSE and R² data are useful for${\;S}_{IO,}$,${\;S}_{LS}$and $S_{CP}$ scenarios, respectively. The FFNN model has the least MAPE and RRMSE, as well as the greatest R² values, demonstrating superior predictive accuracy in seismic design. In addition, it has the quickest computing time (2.4 minutes), which makes it efficient among the networks.

RETRACTED

Seismic Input-Output (S_IO) is a term used to describe the connection between seismic input forces imposed on a structure and the output structural responses that are produced. S_IO is a significant parameter to use in measuring the ability of a model to represent the response of a structure under earthquake loading. Seismic input-output modeling accurately predicts the dynamic response of buildings and other structures to ensure they are safe and perform satisfactorily under seismic loading. Seismic Load-Structure Interaction (S_LS) is the interaction of seismic loads with the structure. This measures the ability of the structure to absorb, transfer, and resist seismic forces depending on the design, material characteristics, and construction techniques. A structure with an optimized seismic load interaction will be able to resist earthquake forces more effectively, minimizing damage and maximizing the resilience of the structure. Seismic Collapse Prediction (S_CP) is a measure of how well a model can predict structural collapse due to seismic loading. S_CP is very important in seismic risk assessment since it assists engineers in establishing the probability of a building or infrastructure collapsing during an earthquake. Collapse prediction is important for designing earthquake-resistant structures and effective retrofitting to improve safety and reduce losses. Coefficient of Determination $R^{2}$is a statistical parameter that tests the goodness of fit of a forecasting model by ascertaining how well the predicted values of the model agree with observed values. A larger $R^{2}$value, nearer to 1, suggests a good fit, i.e., the model efficiently explains variation in the observed data. While doing seismic analysis, a large $R^{2}$value suggests value indicates that the model can predict structural response to earthquake loading accurately, hence the model has significant application in structural engineering and risk assessment.

As Table 2 shows.The proposed FFNN model demonstrates better performance than other methods as shown by the test results of MAPE, RRMSE, R² and computation duration. An FFNN model continuously demonstrates the lowest MAPE values during all scenarios when measuring S_IO (3.0661), S_LS (3.562) and S_CP (3.9252) thereby demonstrating better prediction performance. The proposed FFNN model presents both S_IO (0.0231) and S_LS (0.0281) the lowest RRMSE values which demonstrates precise matching between predicted outcomes and actual observations. The FFNN demonstrates superior performance compared to benchmark models WCFBP-RB, WCFBP-PW1, and WCFBP-MH based on their R² values which reach 1.0096, 1.0995, and 0.9925 for the scenarios. This demonstrates its exceptional explanatory capabilities. The FFNN achieves the tasks within 2.4 minutes while demonstrating its computational effectiveness. The results show that FFNN architecture delivers accurate predictions while requiring less computational resources than other evaluated methods.

RETRACTED

**Table 2:** Outcome of existing and proposed for 6-storey steel structure.

Methods	MAPE			RRMSE			$R^{2}$			Time (min)
	$S_{IO}$	$S_{LS}$	$S_{CP}$	$S_{IO}$	$S_{LS}$	$S_{CP}$	$S_{IO}$	$S_{LS}$	$S_{CP}$	
WCFBP-RB	3.1172	3.679	4.0264	0.0362	0.0394	0.0425	0.9985	0.9983	0.9981	2.7
WCFBP-PW1	3.8244	4.2790	4.7282	0.0485	0.0555	0.0647	0.9921	0.9918	0.9908	2.7
WCFBP-MH	3.5542	3.8993	4.6509	0.0439	0.0512	0.0602	0.9948	0.9936	0.9929	2.5
FFNN (Proposed)	3.0661	3.562	3.9252	0.0231	0.0281	0.0314	1.0096	1.0995	0.9925	2.4

Table 3 summarizes seismic performance for six-story steel structures with varied parameters, including damping coefficient (γ), maximum and minimum wavelengths ($\lambda_{\min}$,$\lambda_{\max}$), and mass. Each item details both the worst and the most effective, and median levels of structural responses, assessed in terms of performance parameters like displacement or stress. Frameworks exhibiting a γ value of 0.02 demonstrate a range of efficiency metrics across numerous wavelength intervals, but those having a γ of 5.00 or 20.0 have considerably higher responses, suggesting significant changes in seismic efficiency depending on attenuation and wavelength. The dataset demonstrates how different settings of λ_min, λ_max and γ values influence structural weight results across 12 testing periods. The weight measurements yield mean results between 9512.12 Kilograms and 9634.30 Kilograms during Trials 1–3 due to the lower γ value of 0.02. When moving from Trials 4–6 with a γ parameter increase from 0.09 to 9411.15 Kg, the mean weights persisted within the range from 9411.15 Kg to 9677.85 Kg which demonstrates average weight efficiency effects. The mean weights show an upward trend at the test condition of γ = 5.00 because Trials 7–9 demonstrate weights between 9801.04 Kg to 9865.02 Kg thus reducing optimization effectiveness. The highest γ value at 20.0 (Trials 10–12) produces further mean weight increase to 9986.58 Kg leading to heavier designs. The trial-to-trial variations of λ_min as well as λ_max simultaneously impact the observed weight fluctuations throughout all trials. Design rates decrease proportionally to lower γ values but higher γ values create heavier less efficient designs during the optimization process thus showing the significance of parameter selection.

RETRACTED

**Table 3:** Sensitivity assessment conducted using PSO for 6-storey.

No	Worst	Weight (Kg)		$\lambda_{\min}$	$\lambda_{\max}$	γ
		Best	Mean			
1	9905.29	9450.50	9612.72	0.0	0.6	0.02
2	9895.40	9461.68	9634.30	0.6	1.5	0.02
3	9797.80	9397.28	9512.12	1.5	2.0	0.02
4	9695.75	9285	9411.15	0.3	0.6	0.09
5	9745.07	9310.72	9677.85	0.4	1.2	0.09
6	9763.12	9436.81	9608.42	1.5	1.0	0.09
7	9845.85	9612.68	9801.04	0.5	1.5	5.00
8	9857.63	9649.53	9865.02	1.0	1.0	5.00
9	9863.82	9635.95	9853.81	1.5	2.0	5.00
10	99672.34	9943.54	9905.45	0.5	1.0	20.0
11	10937.52	9982.01	9945.98	1.0	1.5	20.0
12	11267.50	9994.35	9986.58	1.5	2.0	20.0

Table 4 discusses the design parameters for the seismic study of steel structures using FFNN and PSO are shown in this table. The parameters encompass multiple weight configurations and design limitations for distinct components identified by the labels Q1 through R3. Every entry (Q1, Q2, etc.) provides measurements in the form of W x H (the size x altitude), where ‘W’ stands for width and ‘H’ for height. In addition, the table provides information on the structure’s total weight (9497.32 kg), the total duration (TD) of 2.4 minutes, and data generation time (DGT) of 11.0 minutes. These details are critical for evaluating the stability and performance of the structure during seismic events. The results from PSO+FFNN optimization present a substantially efficient design of the structure. W17 x 35, W17 x 24, and W23 x 65 beam and column sections were chosen because they provide both lightweight performance and structural reliability. The obtained structural weight reached 9497.32 kg as compared to standard baseline weights thus indicating substantial weight reduction. The proposed method demonstrates computational efficiency through its 11.0 minutes design generation time which merges with a total training time of 2.4 minutes. PSO+FFNN executes effectively to determine optimum design parameters alongside quick convergence speed and it becomes a useful tool for structural optimization applications.

**Table 4:** Optimal layouts of 6-storey frames.

Design Parameters	PSO+FFNN (Proposed)
Q1	W17 x 35
Q2	W17 x 24
Q3	W17 x 24
Q4	W23 x65
Q5	W23 x 63
Q6	W23 x 35
R1	W23 x 35
R2	W23 x 35
R3	W11 x24
Weight (kg)	9497.32
DGT (min)	11.0
TT (min)	2.4

Table 5 compares the accuracy of seismic design forecasts for six-story steel structures with two approaches: WCFBP-RB [23] and PSO+FNN (proposed). It compares the expected and actual values of three criteria: seismic input and outcome ($S_{IO}$), the seismic load component ($S_{LS}$), and seismic capacity parameter values ($S_{CP}$). The WCFBP_RB algorithm predicts S_IO_ at 0.6979; however, the actual value is 0.7000, $S_{LS\;}$at 1.3089 versus 1.3491, and $S_{CP}$at 1.9532 instead of 2.0115. The PSO+FFNN technique predicts higher values of $S_{IO}$(0.7879 vs.0.8000), $S_{LS}$(1.4085 vs. 1.4388), and lower $S_{CP}$(1.8621 vs. 1.9000), reflecting a different performance assessment.

RETRACTED

**Table 5:** Performance level in Performance-based seismic design.

Parameter	WCFBP-RB		PSO+FFNN[Proposed]	
	Predicted	Actual	Predicted	Actual
$S_{IO}$	0.6979	0.7000	0.7879	0.8000
$S_{LS}$	1.3089	1.3491	1.4085	1.4388
$S_{CP}$	1.9532	2.0115	1.8621	1.9000

Fig 3 analyses the outcomes of two frameworks, WCFBP-RB [23] and the proposed PSO+FFNN, to forecast three different parameters ($S_{IO,}{\;S}_{LS}$, and${\;S}_{CP}$) to their actual values. This comparison can be represented visually in the form of a graph, featuring an x-axis indicating each parameter and a y-axis indicating their values. Bars or points can indicate the anticipated and actual figures for each parameter, providing for a quick visual evaluation of each design’s accuracy. The graph will show that the PSO+FFNN predictive model’s predictions are often closer to actual values than WCFBP-RB [23], indicating that it may perform better in predicting these parameters.

**Fig 3:** Comparing real and expected <<Eqn143>> max using FFNN (Proposed) for a 6-storey structure.

The IDR comparison of various structural systems emphasizes their seismic behavior and deformation characteristics are shown in Table 6. MRF have the highest drift ratios 1.8% to 3.2%, which are advantageous due to their ductility but need to be designed carefully to avoid excessive deformation. BF provide better stiffness with reduced IDRs (1.2% to 2.5%), thus being more effective in resisting lateral forces. SW exhibit the least drift (0.8% to 1.6%) owing to their stiffness, providing robust lateral resistance. Dual Systems (MRF + SW) provide a balance between strength and ductility, lowering drift (1% to 2%) without compromising on ductility. BI are best, with minimum IDR values (0.5% to 1%) because of their energy dissipation features, making them the best at reducing seismic-induced deformations. In general, although MRF and BF systems are flexible, SW and BI systems are more effective in controlling drift, with Base-Isolation being the most seismic-resistant.

**Table 6:** Comparison of Inter-Story Drift Ratios (IDR) for Different Structural Systems.

Structural System	IDR (S_IO)	IDR (S_LS)	IDR (S_CP)	Max Permissible IDR (%)
Moment-Resisting Frame (MRF)	1.8	2.5	3.2	2.5
Braced Frame (BF)	1.2	1.8	2.5	2.5
Shear Wall System (SW)	0.8	1.2	1.6	2
Dual System (MRF + Shear Wall)	1	1.5	2	2.5
Base-Isolated Structure (BI)	0.5	0.7	1	1.5

As Fig 4 shows.The comparison of structural systems in terms of primary seismic performance criteria discloses huge differences in their seismic resistance. MRF have the largest maximum inter-story drift (2.5%) and residual drift (0.8%), which reflect higher flexibility but also larger post-earthquake deformations. BF present lower values of drift (1.8% max, 0.6% residual) and a greater base shear coefficient (0.15), enhancing lateral load resistance but with a marginally lower energy dissipation efficiency (70%).

RETRACTED

**Fig 4:** Graphical representation of IDR for different structural systems.

As Table 7 shows.SW exhibit very high rigidity, displaying the lowest residual drift (0.3%) and a high base shear coefficient (0.2), with high resistance to seismic forces and attaining 85% energy dissipation efficiency. Dual Systems find a balance, with moderate drift values (1.5% max, 0.5% residual) and high seismic performance (80% energy dissipation).

**Table 7:** Comparison of structural performance based on NRHA results.

Structural System	Max IDR (%)	Residual Drift (%)	Base Shear Coefficient	Energy Dissipation Efficiency	Collapse Probability (%)
MRF	2.5	0.8	0.12	0.75	0.5
BF	1.8	0.6	0.15	0.70	0.3
SW	1.2	0.3	0.2	0.85	0.150
Dual System (MRF + SW)	1.5	0.5	0.18	0.80	0.2
Base-Isolated Structure	0.7	0.1	0.08	0.90	0.50

As Fig 5 shows.BI perform best, with the lowest drift (0.7% max, 0.1% residual), the lowest base shear coefficient (0.08), and the highest energy dissipation efficiency (90%), and with an extremely low collapse probability (0.5%). These observations bring to light that although MRF and BF systems are flexible, SW and Dual Systems are more stable, and Base-Isolation is the most effective in reducing seismic damage.

**Fig 5:** Structural parameters comparison.

As Fig 6 shows.The graph illustrates the accuracy difference between Deep Belief Network (DBN) and Convolutional Neural Network (CNN) along with Deep Convolutional Neural Network (DCNN) through error bars representing the accuracy range. Among the three algorithms the DCNN proves most accurate while CNN ranks second and DBN ranks third. The visual presentation of error bars helps understand result consistency patterns thus showing that although DCNN provides superior average results its variable outcomes need evaluation for practical use. The graphical representation displays an efficient way to understand the reliability and robustness aspects of each model in structural health monitoring operations.

RETRACTED

**Fig 6:** Model performance comparison of DBN, CNN, and DCNN with error bars.

### 4.1 Discussion

The practical deployment of the PSO+FFNN model faces multiple implementation barriers even though it achieves high predictive accuracy along with great efficiency. The process consumes substantial computing resources because users must optimize PSO parameters as well as train the FFNN especially when working with extensive structural optimization problems that have multiple dimensions and complex limitations. To successfully integrate the model within engineering workflows practitioners should perform modifications that fit individual project specifications including project standards and codes. The model’s overall application requires additional testing on authentic datasets to guarantee universal application across various structural plans and seismological events. The acceptance from stakeholders in structural engineering applications of AI-driven solutions depends on making AI models easily interpretable while also requiring ongoing performance checks.

## 5. Conclusion

Study concludes by highlighting a potential method of integrating PSO via FFNN to improve seismic analysis for steel structures. Conversely, to conventional procedures, the technique known as PSO optimizes structural variables and achieves resolution in fewer years, although requiring a large amount of processing power. The FFNN model’s coordination makes it possible to precisely estimate structural reactions, reducing overall computing time. Finally, this combined technique improves structural security and endurance in earthquake scenarios by offering a more accurate and productive process for building seismically resistant steel structures. The suggested FFNN model enhanced MAPE by some 1.6% to 2.5% while lowering RRMSE by around 36% to 46% for all limit states than with the use of the WCFBP-RB method. For R², the new model had relatively similar or a bit higher level, which clearly signifies good forecasting ability. Further, the model showed an improvement in computation time by 11%, further proof of its speed and accuracy as compared to currently available methods.

### Limitations

Study’s limitations include PSO’s high computing cost, which, despite its effectiveness in shrinking centuries, may be excessive for large-scale projects. In addition, while FFNN improves forecast reliability and reduces computation time, its use is dependent on the standard and accessibility of training data, which might restrict its applicability to different structure designs or seismic scenarios.

### Future scope

Future studies could investigate merging sophisticated machine learning algorithms with PSO to enhance seismic design parameters, perhaps enhancing accuracy and computational efficiency. Furthermore, expanding studies to include a wider range of structural morphologies and soil-structure combinations could improve seismic design resilience. Investigating continual monitoring and adaptive design changes during seismic events could also lead to major advances in structural safety.

RETRACTED

## Supporting information

S1 Table FFNN model data. (CSV)

## Abbreviations

PSO: Particles swarm optimization
FFNN: feed-forward neural networks
DBN: Deep belief network
NRHA: Nonlinear Response History Analytics
DCNN: Deep convolutional neural networks
ML: Machine Learning
PBEE: Performance-Based Earthquake Engineering
MAPE: Mean Absolute Percentage Error
WCFBP-RB: Radial Basis Wavelet Cascade-Forward Back Propagation
SHM: Structural Health Monitoring
WCFBP-PW1: Polynomial Wavelet 1 Wavelet Cascade-Forward Back Propagation
RRMSE: Relative Root Mean Squared Error
CNN: Convolutional Neural Network
DGT: Data Generation Time
WCFBP-MH: Wavelet Cascade-Forward Back Propagation with Morlet Wavelet
TT: Total Times
RID: Remnant Interstory Drift
$S_{IO}$: Immediate Occupancy with S parameter
$S_{LS}$: Life Safety with S parameter
$S_{CP}$: Collapse Prevention with S parameter
